# Clinical Effect of Metronidazole Vaginal Effervescent Tablet Combined with Flavescentis Sophora Suppository in the Treatment of Trichomonas Vaginitis

This article has been retracted.

**DOI:** 10.1155/2022/1250755

**Published:** 2022-08-04

**Authors:** Lingjia Shi, Dan Yang, Xin Wang

**Affiliations:** ^1^Gynaecology, Shaoxing City Keqiao District Hospital of Traditional Chinese Medicine, Shaoxing 312030, China; ^2^Department of Rehabilitation, Huai'an Second People's Hospital, The Affiliated Huaian Hospital of Xuzhou Medical University, Huai'an 223002, China; ^3^Endocrine Department, Lianshui People's Hospital Affiliated to Kangda College of Nanjing Medical University, Lianshui 223400, China

## Abstract

For the treatment of trichomonas vaginitis, a combination therapy of metronidazole vaginal effervescent tablet combined with Flavescentis Sophora suppository is proposed. The patients diagnosed with trichomonas vaginitis are divided into the conventional treatment group and the joint group. The conventional group is treated with metronidazole vaginal effervescent tablets, and the joint group is treated with metronidazole vaginal effervescent tablets combined with sophora bolt. Both groups are treated for 3 months to observe the therapeutic effect of the two treatment methods. The expressions of IL-2 and IL-13 in serum of patients are detected by the ELISA. The changes in the vaginal pH value and cleanliness at each time point are observed. The patients are followed up for 6 months after treatment in order to observe the recurrence of trichomonas vaginitis in both groups. Experimental results show that the combination of the two tablets can further improve the clinical efficacy and reduce the inflammatory response and effectively improve the PH value and cleanliness of the vagina, and the recurrence rate is lower, which is worthy of clinical application.

## 1. Introduction

Trichomonal vaginitis, as a gynecological disease often occurring in women of childbearing age, is mainly caused by vaginal pH imbalance caused by trichomonad infection, which leads to vaginitis. Without timely intervention and treatment, it may further develop precancerous lesions, cause infertility and other symptoms, and pose a serious threat to women's life and health [1, 2]. Incomplete statistics show that the incidence of sexual vagina trichomonad disease is on the rise year by year, and such diseases with high infectivity, clinical symptoms of vaginal ectopic, itching, leucorrhoea increase, etc., and if treatment is not in place, there will be a relapse, greatly increased the psychological pressure and reduce the quality of life in patients [3]. Therefore, it is of great significance to find a safe and effective treatment to improve the prognosis and quality of life of patients with trichomoniasis vaginitis [4].

Metronidazole vaginal effervescent tablet is a common way to treat trichomonas vaginitis in clinical practice, which can inhibit the growth of anaerobic bacteria and trichomonas, while Flavescentis Sophora suppository, as a Chinese medicine composed of Flavescentis Sophora total alkali, lanolin, and semisynthetic fatty acid ester, has certain antibacterial and anti-inflammatory effects [5, 6]. However, there are relatively few studies on the combination of the two methods in the clinical treatment of trichomonal vaginitis, and based on the study by choosing 98 cases of patients with trichomonas vaginitis, we adopt different treatments and we observe the clinical curative effect of metronidazole vaginal effervescent tablets combined with sophora bolt for the treatment of trichomonas vaginitis which provides a new theoretical basis for treatment.

The rest of this paper is organized as follows: Section 2 discusses related work, followed by the treatment methods and efficacy evaluation for treatment of trichomonas vaginitis designed in Section 3.  Section 4 is the technology roadmap and statistical processing.  Section 5 shows the experimental results for comparison of treatment efficiency, and Section 6 concludes the paper with summary and future research directions.

## 2. Related Work

Trichomonas vaginitis, a common type of vaginitis in women, is mainly caused by *Trichomonas vaginalis* and is a high susceptibility and infectious disease, with clinical manifestations of vaginal itching, more increased leucorrhoea, and appearance of the symptoms such as foam. Severe cases can lead to precancerous lesions and also greatly interfere with the normal life and the life and health of patients [7, 8]. *Trichomonas vaginalis*, a flagellate, will interfere with normal vaginal glycogen and destroy the immune defense system of the vagina itself, resulting in low vaginal immune function, and the vagina will be subsequently infected by a variety of bacteria; it can easily cause recurrence without radical treatment [9]. In pregnant women, at the same time, *Trichomonas vaginalis* may hinder the vagina's lactic acid secretion which affects the survival rate of the sperm in the vagina, causing infertility symptoms; therefore, seeking a safe, highly effective, and radical treatment for improving the prognosis of patients with trichomonas vaginitis and improving the quality of life is of great significance [10].

Metronidazole vaginal effervescent tablets, one of the nitroimidazole derivatives, can inhibit the redox reaction of amoeba and break the nitrogen chain of the protozoa. In addition, because metronidazole has the effect of antianaerobic bacteria and antigen-flushing, it can be used in clinical treatment of a variety of infections caused by anaerobic bacteria [11]. At the same time, metronidazole vaginal effervescent tablets can be rapidly absorbed and widely reached into various tissues and body fluids through vaginal administration and can effectively cross the blood-brain barrier and can be distributed in various body fluids, giving play to their anti-inflammatory and anti-insect effects [12]. As a kind of traditional Chinese medicine suppositories, oxymatrine and other alkaloids in the suppositories can play antibacterial, drudgery, and insecticidal roles in the body. Zhang [13] also indicated that the oxymatrine suppositories could enhance immunity after being absorbed by the body and effectively inhibit the proliferation of *Trichomonas*. In addition, Flavescentis Sophora suppository also has the characteristics of quick acting, which is absorbed by the vaginal mucosa in a short time after being inserted into the vagina, and its ingredients are all Chinese medicinal materials with relatively few toxic and side effects [14].

## 3. Treatment Methods and Efficacy Evaluation

A retrospective analysis was performed on 98 patients diagnosed with trichomoniasis vaginitis in our hospital from August 2020 to August 2021 who were divided into the conventional group (*n* = 49) and combined group (*n* = 49) according to different treatment methods. The comparison of the baseline data between the two groups is shown in Table 1, showing comparability (*P* > 0.05). All patients included in the study have the right to know and consent to the treatment adopted and fully understand the possible adverse reactions after medication. The clinical data and general information collected in this study are kept confidential and will not be used for other purposes.

The inclusion criteria mainly include four aspects:(1) all patients met the clinical diagnostic criteria for trichomoniasis vaginitis [15]; (2) good treatment compliance; (3) complete general information and clinical data; (4) good communication and understanding skills.

The exclusion criteria mainly include four aspects:(1) accompanied by mental diseases, unable to cooperate with the study; (2) have a history of allergy to the drugs used in this study; (3) lost contact during follow-up; (4) unauthorized use of other drugs during treatment resulted in deviation of research results [16].

### 3.1. Treatment Methods

The conventional group was treated with metronidazole vaginal effervescent tablets (manufacturer: Jilin AodongYanbian Pharmaceutical Co., LTD., specification: 0.2 g, Batch No.: National Medicine Approval: H22020774), and 0.2 g metronidazole vaginal effervescent tablets were injected every night before going to bed.

The combined group was treated with matrine suppositories (manufacturer: Shaanxi Dongtai Pharmaceutical Co., LTD., specification: 6 pills/box, Batch No.: National Medicine Approval Z20053241) on the basis of the conventional group. The matrine suppositories were put into the deep vulva after washing clothes before going to bed, once a day, once a time. Both groups were treated for 3 months and followed up for 6 months after treatment.

### 3.2. Enzyme-Linked Immunosorbent Assay for IL-2 and IL-13

At each time point before and after treatment, 5 ml of fasting venous blood was taken from the patients in the morning and centrifuged for 10 min at a speed of 3500 r/min. The supernatant was taken after centrifugation, and serum IL-2 and IL-13 were detected by the ELISA. The kits were purchased from Shanghai Enzyme-linked Biotechnology Co., LTD, and the instructions in the kit were followed.

### 3.3. Detection of Vaginal pH and Vaginal Cleanliness

At each time point before and after treatment, a glass stick was used to dip an appropriate amount of vaginal secretions and smear it evenly on the pH test paper. The changes in vaginal pH were read against the standard color card.

The vaginal secretion wet film and stained smear were observed under an electron microscope, and the cleanliness degree of the vagina was divided into four grades. Grade 1: under the microscope, the main bacteria in the vagina were vaginal bacillus, and a large number of epithelial cells could be observed; grade 2: there are a few pus cells and miscellaneous bacteria in the vagina under the microscope; grade 3: the number of pus cells and miscellaneous bacteria under the microscope was significantly more than that of vaginal bacillus and epithelial cells; grade 4: microscopic results showed that the patient's secretions were almost all pus cells and miscellaneous bacteria, and almost no vaginal bacteria and epithelial cells existed. Grades 1 to 4 were marked as 1 to 4 points respectively, and the higher the score was, the worse the cleanliness of the patient's vagina was.

### 3.4. Efficacy Evaluation

According to the following criteria, the clinical efficacy was divided into cured, significant effect, effective, and ineffective, among which all clinical symptoms disappeared after treatment; the culture results of trichomonas were negative, and the cleanliness of the vagina was grade 1, which was classified as cured. The clinical symptoms were significantly relieved after treatment, and the negative culture results of trichomonas and vaginal cleanliness ≤2 were considered significant effects. Clinical symptoms and vaginal cleanliness were slightly improved after treatment, and the trichomonas culture results were weakly positive and classified as effective. No changes in clinical symptoms, vaginal cleanliness, and trichomonas culture results after treatment were classified as ineffective. Clinical effective rate = (cure + significant effect + effective)/number of people × 100%.

## 4. Technology Roadmap and Statistical Processing

### 4.1. Technology Roadmap

Figure 1 shows the technology roadmap of this study.

### 4.2. Statistical Processing

All data during the study were collected and sorted and put into SPSS22.0 for statistical processing. If the measurement data followed normal distribution and homogeneity of variance, they were expressed as the mean ± standard deviation. The intergroup differences were performed by the independent sample *T* test, intragroup comparison was performed by the paired *T* test, repeated measurement analysis was performed between different time points, and the spherical test was performed. Counting data were represented by *N* (%), and the difference between groups was tested by the *X*2. Kaplan–Meier survival curve was used to observe the recurrence of trichomonas vaginitis [17–19]. All the above data were statistically significant at *P* < 0.05, and the differences among the data were statistically significant.

## 5. Experimental Results

### 5.1. Comparison of Treatment Efficiency between the Two Groups

After 3 months of treatment, the overall effective rate of the combined group was significantly higher than that of the conventional group (*P* < 0.05), as shown in Table 2.

### 5.2. Changes of IL-2 and IL-13 at Different Time Points

Table 3 and Figure 2 show the expression of IL-2 in each group, and Table 4 and Figure 3 show the trend of IL-13. In Table 3, “^*∗*^” means that compared with T1, ^*∗*^*P* < 0.05, “#” indicates that compared with T2, ^#^*P* < 0.05, and “&” means ^&^*P* < 0.05 compared with T3. In Table 4, “^*∗*^” means that compared with T1, ^*∗*^*P* < 0.05. “#” indicates that compared with T2, ^#^*P* < 0.05. “&” means ^&^*P* < 0.05 compared with T3. In Figures 2 and 3, “a, b, c, d” means that if the same letter is shared between groups, *P* > 0.05 at different time points. “#” indicates that *P* < 0.05 between the two groups compared at the same point.

Before treatment, there was no difference in the expression of IL-2 and IL-13 in the two groups, but after certain treatment, the expression of all inflammatory factors decreased, and the inflammatory factors in the combined group were lower than those in the conventional group at each time point after treatment (all *P* < 0.05).

### 5.3. Observing the Changes of the Vaginal pH Value and Cleanliness at Each Time Point

The groups of vaginal pH expression changes are shown in Table 5 and Figure 4, the vaginal cleanness trends are shown in Table 6 and Figure 5, and the vaginal PH value and cleanliness of the two groups before treatment have no difference. But after a certain treatment of each index declined, after treatment, improved indicators of the joint group at all-time points are better than those of the conventional group (all *P* < 0.05). In Tables 5 and 6, “^*∗*^” means that compared with T1, ^*∗*^*P* < 0.05; “#” indicates that compared with T2, ^#^*P* < 0.05; “&” means ^&^*P* < 0.05 compared with T3. In Figures 4 and 5, “a, b, c, d,” respectively, means that if the same letter is shared between groups, *P* > 0.05 at different time points. “#” indicates that *P* > 0.05 between the two groups compared at the same point.

### 5.4. Comparison of the Incidence of Adverse Reactions after Treatment

There was no difference in adverse reactions between the two groups after treatment (*P* > 0.05), as shown in Table 7.

### 5.5. Kaplan–Meier Survival Curve

The Kaplan-Meier survival curve is drawn to observe the recurrence of trichomonas vaginitis. The survival curve results showed that the recurrence rate of the conventional group was significantly higher than that of the combined group after 6 months of treatment (*x*^2^ = 5.145, *P*=0.023), as shown in Figure 6.

## 6. Conclusion

The results in this paper show that the clinical effective rate of matrine suppositories combined with metronidazole vaginal effervescent tablets was significantly higher than that of metronidazole effervescent tablets alone, suggesting that both drugs have anti-inflammatory, bactericidal, and anti-insect effects, so the combination of two drugs can further enhance the efficacy and improve the clinical effective rate. In addition, compared with the conventional group, the combined group had lower levels of IL-2 and IL-13 after treatment. Both IL-2 and IL-13, as interleukins, act as lymphatic factors between white blood cells and immune cells and participate in hematopoietic and immune regulation together with blood cells and play an important role in regulating inflammation. The increase in their expression level in the body indicates the occurrence of inflammatory response in the body and the imbalance of immune regulation function, and the combination treatment of the two drugs can further reduce the level of inflammatory factors, indicating that its anti-inflammatory effect is significantly enhanced compared with the single drug. In addition, the comparison of the vaginal pH value and cleanliness before and after treatment showed that the combination of drugs has a more significant effect on improving the vaginal microenvironment, which can further maintain the balance of vaginal pH and reduce the number of pus cells and miscellaneous bacteria, which is conducive to further recovery of the disease. By comparing the results of adverse reactions after therapy, we found that two ways illustrate that they have higher security, but the Kaplan– Meier survival curve shows combination can further reduce the recurrence rate, to improve the prognosis of trichomonas vaginitis patients, and has more significant effects.

Above all, compared to a single use of metronidazole vaginal effervescent tablets for trichomonas vaginitis, the combination of sophora bolt strengthened clinical efficacy and can significantly decrease the body's inflammatory response and further restore vaginal pH balance, keep the vagina clean, and ensure lower recurrence rate after treatment; However, the safety of the two groups is very high, and the combination of drugs is more recommended for the treatment of trichomonal vaginitis.

## Figures and Tables

**Figure 1:** Technology roadmap of this study.

**Figure 2:** The trend of IL-2 changes.

**Figure 3:** The trend of IL-13 changes.

**Figure 4:** Vaginal pH changes.

**Figure 5:** Vaginal cleanliness changes.

**Figure 6:** Comparison of recurrence rates.

**Table 1:** The baseline data.

	Conventional group (*n* = 49)	Combined group (*n* = 49)	*t/x * ^2^	*P*
Age (years)	34.42 ± 7.63	34.17 ± 7.58	0.163	0.871
BMI (kg/m^2^)	23.33 ± 2.15	23.25 ± 2.14	0.185	0.854
Course of the disease (month)	11.15 ± 3.36	11.21 ± 3.28	−0.089	0.929
Level of education				
Primary and below	12 (24.49%)	11 (22.45%)	2.363	0.732
Junior to senior high	28 (57.14%)	30 (61.22%)		
University and above	9 (18.37%)	8 (16.33)		

**Table 2:** Therapeutic response rate.

Group	*n*	Cured	Significant effect	Effective	Ineffective	Effective rate
Combined group	49	18 (36.73%)	21 (42.86%)	7 (14.29%)	3 (6.12%)	46 (93.88%)
Conventional group	49	7 (14.29%)	17 (34.69%)	15 (30.61%)	10 (20.41%)	39 (79.59%)
*x * ^2^						4.346
*P*						0.037

**Table 3:** The trend of IL-2 changes.

Group	*n*	*T*1	*T*2	*T*3	*T*4	*F*	*P*
Combined group	49	9.34 ± 2.19	7.22 ± 1.98^*∗*^	6.18 ± 1.63^∗#^	5.24 ± 1.25^∗#&^	6.642	＜0.001
Conventional group	49	9.32 ± 2.17	8.23 ± 2.05^*∗*^	7.64 ± 1.87^*∗*^	6.64 ± 1.67^∗#&^	4.451	0.003
*t*		0.045	−2.481	−4.120	−4.698		
*P*		0.964	0.015	＜0.001	＜0.001		

**Table 4:** The trend of IL-13 changes.

Group	*n*	*T*1	*T*2	*T*3	*T*4	*F*	*P*
Combined group	49	36.66 ± 3.19	30.22 ± 2.74^*∗*^	24.42 ± 2.53^∗#^	20.16 ± 2.15^∗#&^	7.723	＜0.001
Conventional group	49	36.63 ± 3.25	32.74 ± 2.86^*∗*^	29.35 ± 2.78^∗#^	26.63 ± 2.32^∗#&^	5.624	＜0.001
*t*		0.046	−4.454	−9.181	−14.318		
*P*		0.963	＜0.001	＜0.001	＜0.001		

**Table 5:** The changing trend of the vaginal pH value.

Group	*n*	*T*1	*T*2	*T*3	*T*4	*F*	*P*
Combined group	49	6.93 ± 0.63	5.63 ± 0.53^*∗*^	4.57 ± 0.43^∗#^	3.82 ± 0.27^∗#&^	5.532	＜0.001
Conventional group	49	6.91 ± 0.61	6.03 ± 0.56^*∗*^	5.34 ± 0.53^∗#^	4.93 ± 0.31^∗#&^	3.326	0.034
*t*		0.160	−3.631	−7.897	−18.901		
*P*		0.873	＜0.001	＜0.001	＜0.001		

**Table 6:** The changing trend of vaginal cleanliness.

Group	*n*	*T*1	*T*2	*T*3	*T*4	*F*	*P*
Combined group	49	2.73 ± 0.56	2.12 ± 0.42^*∗*^	1.78 ± 0.33^∗#^	1.21 ± 0.29^∗#&^	4.426	＜0.001
Conventional group	49	2.72 ± 0.58	2.33 ± 0.48^*∗*^	2.04 ± 0.42^∗#^	1.98 ± 0.32∗^#^	3.325	0.028
*t*		0.087	−2.305	−3.407	−12.481		
*P*		0.931	0.023	0.001	＜0.001		

**Table 7:** Adverse reaction comparison.

Group	*n*	Nausea and vomiting	Bad breath	Diarrhea	Rash	Occurrence rate
Combined group	49	4	3	1	3	11 (22.45%)
Conventional group	49	3	2	2	1	8 (16.33%)
*x * ^2^						0.588
*P*						0.443

## Data Availability

The simulation experiment data used to support the findings of this study are available from the corresponding author upon request.
